# Comparison of Conventional Modeling Techniques with the Neural Network Autoregressive Model (NNAR): Application to COVID-19 Data

**DOI:** 10.1155/2022/4802743

**Published:** 2022-06-14

**Authors:** Muhammad Daniyal, Kassim Tawiah, Sara Muhammadullah, Kwaku Opoku-Ameyaw

**Affiliations:** ^1^Department of Statistics, Islamia University of Bahawalpur, Bahawalpur, Pakistan; ^2^Department of Mathematics and Statistics, University of Energy and Natural Resources, Sunyani, Ghana; ^3^Department of Statistics and Actuarial Science, Kwame Nkrumah University of Science and Technology, Kumasi, Ghana; ^4^Pakistan Institute of Development Economics, Islamabad, Pakistan; ^5^National Institute of Health, Islamabad, Pakistan

## Abstract

The coronavirus disease 2019 (COVID-19) pandemic continues to destroy human life around the world. Almost every country throughout the globe suffered from this pandemic, forcing various governments to apply different restrictions to reduce its impact. In this study, we compare different time-series models with the neural network autoregressive model (NNAR). The study used COVID-19 data in Pakistan from February 26, 2020, to February 18, 2022, as a training and testing data set for modeling. Different models were applied and estimated on the training data set, and these models were assessed on the testing data set. Based on the mean absolute scaled error (MAE) and root mean square error (RMSE) for the training and testing data sets, the NNAR model outperformed the autoregressive integrated moving average (ARIMA) model and other competing models indicating that the NNAR model is the most appropriate for forecasting. Forecasts from the NNAR model showed that the cumulative confirmed COVID-19 cases will be 1,597,180 and cumulative confirmed COVID-19 deaths will be 32,628 on April 18, 2022. We encourage the Pakistan Government to boost its immunization policy.

## 1. Introduction

One of the brutal pandemics in human history, coronavirus disease 2019 (COVID-19), has caused millions of human fatalities around the world and continues to rage havoc worldwide since its outbreak in 2019. The pandemic has reshaped scientific thinking and study. Scientists around the world continue to study various variants of this deadly disease to devise strategies to eliminate it from the human race. The different variant of the virus has made it even more hectic for vaccine manufacturers. Vaccinated individuals even get infected with the virus but with a lower risk of dying compared to the unvaccinated [1, 2]. Numerous modeling and forecasting techniques have been proposed for COVID-19 confirmed cases and deaths.

Anwar and Mokhtar [3] utilized an Epidemic Calculator that uses a susceptible, exposed, infected, and recovered (SEIR) compartmental model with information from the Egyptian Ministry of Health and Population. For the most elevated assessed case mortality rate (7.7%), the number of individuals admitted in hospitals was anticipated to top in the middle of June, with a sum of 20,126 in the hospitals and an anticipated death total of 12,303. Statistical modeling and machine learning techniques were applied to foresee and gauge the completion phase of COVID-19 utilizing different time contamination rates and individual numbers of contacts [4, 5]. Their outcomes indicated that the assessed generation number was 2.2 in Kuwait, with the contact rate among the populace on the high side, denoting an epidemic top value unlikely to be reached and the nation requiring a more severe mediation course of action.

El Desouky [6] forecasted the pinnacle, duration, and reenactment of possible varieties that may be occurring in the social ways and behavior of Egyptians in the sacred season of Ramadan. They recommended three perceived numerical methods (i.e., Euler's method and Runge Kutta method of request two (RK2) and of request four (RK4)) for tackling such conditions of health care globally and subsequently making significant sources of information available. Benkouiten et al. [7] were optimistic that Hajj pilgrims played a key role in the dispersion of the pandemic. Numerical outcomes might be utilized to figure out the number of vulnerable persons to the disease, recuperated, and isolated persons in the long run to help unfamiliar endeavors to develop their mediation benefits and further anticipation. Numerical methodologies and calculated models [8, 9] have been utilized for analyses and understanding of COVID-19.

Pirouz et al. [10] concentrated on the arrangement of confirmed instances of COVID-19 utilizing an Artificial Intelligence (AI) strategy, local area information steering arrangement of the neural network, by adapting a twofold characterization modeling. The proposed model depends on a contextual analysis of China's Hubei territory. A few significant parameters like greatest daily temperature, least daily temperature, normal day-to-to-day temperature, density, relative density, and speed of the wind as well as the quality of the air [11] were parsed as the informational index and picked the number of affirmed cases as the result of information collection for thirty days. They were of the view that the parallel order model gives more prominent ability to exactness in anticipating the announced cases. Besides, they played out the relapse analysis and the example of revealed cases relative to the variety of everyday climatic conditions (speed of the wind, relative density, and normal temperature). Their outcome pointed out that the relative density and the most extreme everyday temperature greatly affected the actual cases. The examination of the observed confirmed COVID-19 cases using machine learning approaches revealed that the variable number of tests in a particular country did not assume any crucial part in the expectation of the aggregate number of confirmed cases [12]. Pham et al. [13] provided a new AI version and a large data application to properly comprehend the situation of COVID-19 and provided alternatives in ceasing COVID-19 outburst to manage the viral mutation spread.

Ranjan [14] compared data on the COVID-19 upsurge in India and multiple countries together with key counties in the United States (US) and noted that India's first number of reproductions, *R*_0_, is anticipated to be around 1.4 × 10^3.9^. At the time, the growth ring of India's infection and that of Washington and California were close. Traditional and integrated models of susceptible-infected-recovered (SIR) model, depending on the data recently organized, were applied to render a recurring short-ring and long-term prognosis. The SIR model estimated India's stability by the end of May, 2020, with a proposed final size of the epidemic around 13,000, although the approximation will be invalid in the instance that India enters the group transmission point. By the application of a similar model, Italy was assumed to reach its pandemic peak on March 21, 2020 [15].

Admittance to real-time information and the powerful use of episode expectation or estimating models are central to getting quick data with respect to the transmission elements of the infection and its ramifications. Besides, every flare-up has novel transmission qualities that are unique in relation to different episodes, which brings up the issue of how standard expectation models would act in delivering precise outcomes. Moreover, different elements including the number of known and obscure factors, contrasts in populace/behavioural intricacies in different geopolitical regions, and variety in control procedures influence the vulnerability of forecast models [16]. Thus, it is challenging for standard epidemiological models like susceptible-infected-recovered (SIR) to give reliable outcomes to long-haul forecasts. Hence, it is vital to not just review the relationship between the parts of the episode data sets but also evaluate the adequacy of the normal sickness expectation models.

As of late, there have been a handful of works that attempt to understand the spread of COVID-19 as well as predict confirmed cases and deaths of COVID-19, especially making use of statistical methodologies. For example, Kucharski et al. [17] investigated a blend of stochastic transmission models on four data sets that caught the everyday number of new cases, the day-to-day number of new internationally sent out cases, the extent of contaminated travelers on departure flight, and the quantity of new confirmed cases to appraise the transmission elements of the illness throughout some time [18]. Machine learning-based model has been applied to analyze and predict the growth of COVID-19 [19]. Guo and He [20] utilized AI to predict cases and deaths attributed to COVID-19 globally. Models of the Markov chain have been availed to predict COVID-19 spread based on secondary data as of March 13, 2020. Xu et al. [21] and Arumugam and Raji [22] utilized Markov models to predict the impact of the coronavirus on the human race using probability matrices and Monte Carlo simulation. Bertozzi et al. [23] opined that the COVID-19 pandemic has put epidemic modeling at the lead of international public policy making.

Al-qaness et al. [24] put forward an updated version of the adaptive neuro-fuzzy inference system (ANFIS) applying an amplified flower pollination algorithm (FPA) after implementing the salp swarm algorithm (SSA). Wu et al. [25] deduced that the COVID-19 epidemic is now filling dramatically in different significant urban areas of China with a fall time behind the Wuhan episode of around one to fourteen days using the susceptible-exposed-infectious-recovered metapopulational model in a Markov Chain Monte Carlo framework. A blended nonlinear assessment approach consolidating the Gaussian process (GP) and unscented Kalman filter (UKF) was suggested to anticipate the dynamic changes in wind speed and further develop the forecasting accuracy [26]. Zhao et al. [27] predicted new COVID-19 cases in a US state using Poisson and gamma distributions. Hao et al. [28] utilized the advancement pattern investigation of confirmed COVID-19 cumulative cases, cumulative deaths, and cumulative recovered cases in Wuhan from January 23, 2020, to April 6, 2020, by implementing an Elman neural network, long short-term memory (LSTM), and support vector machine (SVM) for future predictions.

Time-series models have been broadly applied to COVID-19 data. Tawiah et al. [29] proposed zero-inflated time-series model for COVID-19 deaths in Ghana. Luo et al. [30] used LSTM and XGBoost algorithms to predict COVID-19 transmission in America using time series. Gecili et al. [31] forecasted COVID-19 confirmed deaths, recovery, and cases in the USA and Italy through the application of novel time-series modeling. Barría-Sandoval et al. [32] predicted COVID-19 cases in Chile by employing time-series techniques. Chyon et al. [33] applied machine learning techniques to autoregressive integrated moving average (ARIMA) models [34] to predict COVID-19 cases. Ali et al. [35] suggested that ARIMA models are suitable for epidemic forecasting. Doornik et al. [36] depicted how to disintegrate the detailed time series of COVID-19 confirmed cases and deaths into a trend, seasonal, and irregular component utilizing machine learning approaches. Nevertheless, forecasting and modeling escalation of COVID-19 persist as a challenge. Therefore, other time-series methods can be explored to forecast confirmed COVID-19 cases and deaths.

In the time-series domain, improving forecasting accuracy is an important and often tricky task confronting data analysts in different areas. Although many time-series models are available in the literature, the study for boosting the ability of prediction models has never stopped. In this paper, we model and forecast the confirmed cumulative COVID-19 cases and deaths in Pakistan based on Box–Jenkins time series, ARIMA model, and neural network autoregressive (NNAR) model vis-a-vis other competing models, thereby comparing them. The proposed model forecast will go a long way to help authorities to develop new strategies to combat the pandemic in Pakistan.

In the subsequent sections of the paper, we present the materials and methods applied, the results, and discussion of the statistical modeling vis-a-vis the conclusions of the study.

## 2. Materials and Methods

### 2.1. Data

The data used in this study consist of new confirmed COVID-19 cases and deaths in Pakistan from the first reported case on February 26, 2020, to February 18, 2022, provided by the COVID-19 Health Platform of the Ministry of National Health Services Regulation, Government of Pakistan. We utilized cumulative data on the confirmed cases and deaths. It can be noted from Figure 1 that the cumulative cases and deaths show exponential growth with respect to time, so nonseasonal ARIMA modeling can be used to forecast the trend of current COVID-19 cases and deaths. The summary statistics of the data used in the study are presented in Table 1. It can be observed that the average daily confirmed COVID-19 cases were 2064, and the average daily deaths attributed to COVID-19 were 41 from February 26, 2020, to February 18, 2022. The minimum daily confirmed cases and daily deaths were 0, respectively, while the maximum confirmed daily cases were 8183 and the maximum daily death was 313.

### 2.2. Methods

The Box–Jenkins ARIMA (*p*, *d*, *q*) [37] is given by

(1) $$\begin{array}{c} {\hat{X}}_{t}=\mu +\alpha_{1}{\hat{X}}_{t-1}+\cdots +\alpha_{p}{\hat{X}}_{t-p}+\cdots +\theta_{1}\epsilon_{t-1}+\cdots +\theta_{q}\epsilon_{t-q}+\epsilon_{t}, \end{array}$$

where $\alpha_{1}{\hat{X}}_{t-1},\ldots ,\alpha_{p}{\hat{X}}_{t-p}$ are the lagged values and *θ*_1_*ϵ*_*t*−1_,…, *θ*_*q*_*ϵ*_*t*−*q*_  are the lagged errors of the series ${\hat{X}}_{t}$. The constants *p*, *d* and *q* represent the order of the autoregressive term, the degree of differencing series, and the order of the moving average term, respectively. *ϵ*_*t*_ is the white noise with mean 0 and variance *σ*^2^. ${\hat{X}}_{t}$ can be differenced once or more.

The Box–Jenkins multiplicative seasonal ARIMA model [37–40] represented by ARIMA (*p*, *d*, *q*) × (*P*, *D*, *Q*) is given by

(2) $$\begin{array}{c} \beta_{p}\left(K\right)\gamma_{P}\left(K^{f}\right){\left(1-K\right)}^{d}{\left(1-K^{f}\right)}^{D}{\hat{X}}_{t}=\omega +\alpha_{q}\left(K\right)\varphi_{Q}\left(K^{f}\right)\epsilon_{t}, \end{array}$$

with *β*_*p*_(*K*)=1 − *β*_1_*K* − ⋯*β*_*p*_*K*^*p*^; *γ*_*P*_(*K*^*f*^)=1 − *γ*_1_*K*^*f*^ − ⋯−*γ*_*P*_*K*^*Pf*^;  *α*_*q*_(*K*)=1 − *α*_1_*K* − ⋯*α*_*q*_*K*^*q*^;  and *φ*_*Q*_(*K*^*f*^)=1 − *φ*_1_*K*^*f*^ − ⋯−*φ*_*Q*_*K*^*Qf*^, where *K* is the operator balanced shift and *f* is the frequency of seasonality. *D* and *d* are the seasonal difference and ordinary differencing degrees, respectively. *β*_*p*_(*K*) and *γ*_*P*_(*K*^*f*^) are the regular autoregressive polynomial of order *p* and seasonal autoregressive polynomial of order *P*, respectively. Also, *α*_*q*_(*K*) and *φ*_*Q*_(*K*^*f*^)  are the polynomials of regular moving average of order *q* and seasonal moving average of order *Q*, respectively. Similarly, *ω*=*ρ*(1 − *β*_1_ − ⋯*β*_*p*_)(1 − *γ*_1_ − ⋯−*γ*_*P*_), where the mean of the process ${\left(1-K\right)}^{d}{\left(1-K^{f}\right)}^{D}{\hat{X}}_{t}$ is *ρ*. *ϵ*_*t*_ is the white noise with mean 0 and variance *σ*^2^.

Shunway and Stoffer [38] proposed that to maintain casualty and investibility, the solution set of all polynomials in the multiplicative model must be outside the unit circle. For simplicity, we assumed *ω*=0. Thus, we selected the most apt values of *p*, *d*, *q*, *P*, *D*, and *Q* by calculating and examining the autocorrelation function (ACF) and the partial autocorrelation function (PACF) of our data by graphing the time series and identifying any unusual data points as well as selecting the appropriate transformation of the variance stabilization. We determined the order of *p*, *q*, *P*, and *Q* by the examination of the ACF and PACF [41]. We employed the portmanteau test for the residual analysis to check for autocorrelation. For an adequate model, the errors are expected to be uncorrelated or white noise [42]. The portmanteau test confirms the ACF residual plots, PACF residual plot, and the normal probability plot.

The model with the least root mean square error (RMSE) and mean absolute error (MAE) is selected as the most appropriate for our data. The expressions RMSE and MAE are

(3) $$\begin{array}{c} \text{RMSE}=\sqrt{\frac{1}{T-N}\sum_{t=N+1}^{T}{\left(X_{t}-{\hat{X}}_{t}\right)}^{2}},\\ \text{MAE}=\frac{1}{T-N}\sum_{t=N+1}^{T}\left|X_{t}-{\hat{X}}_{t}\right|, \end{array}$$

where *X*_1_,…,  *X*_*N*_ and *X*_*N*+1_,…, *X*_*T*_ are the partitions of the data. These metrics summarize as well as assess the quality of the model. The smaller the value, the better the model with a superior quality for forecasting.

We used the Dickey–Fuller (DF) test, the Phillips–Perron (PP) test, and Augmented Dickey–Fuller (ADF) test, which are unit root tests, to check whether our data are stationary or not. Violations were corrected to meet all necessary assumptions of the model.

#### 2.2.1. Neural Network Autoregressive Modeling

We focused on the NNAR model with a hidden layer selected automatically throughout the modeling process. Lagged values of the time series can really be employed as input data to a neural network with time-series data, exactly as it is done with lagged values in a linear autoregressive model. When this is done, the model is referred to as an NNAR model. An NNAR (*p*, *kp*, *k*) denotes the hidden layer has *pp* delayed inputs and *kk* nodes. Moreover, NNAR (*p*, 0*p*, 0) model is the same as an ARIMA (*p*, 0*p*, 0) but without parameter limitations that assure stationarity. The NNAR (*p*, *kp*, *k*) [43, 44] is represented by

(4) $$\begin{array}{c} f\left(X\right)=\beta_{0}+\sum_{k=1}^{K}\beta_{k}g\left(w_{k0}+\sum_{j=1}^{p}w_{kj}X_{j}\right). \end{array}$$

The expression is constructed in two stages. The *K* activations come first. In the activation, *A*(*k*), *k*=1,   …, *K*, the hidden layer is calculated as a function of the input characteristics *X*_*j*_=*X*_*t*−1_,…, *X*_*t*−*p*,_  with

(5) $$\begin{array}{c} A\left(k\right)=h\left(k\right)=g\left(w_{k0}+\sum_{j=1}^{p}w_{kj}X_{j}\right), \end{array}$$

where *g* is a previously defined nonlinear activation function. Each *A*(*k*) may be seen as a separate *h*_*k*_(*X*) transformation of the unique characteristics. The output layer receives these *K* instigations from the hidden layer.

(6) $$\begin{array}{c} f\left(X\right)=\beta_{0}+\sum_{k=1}^{K}\beta_{k}A\left(k\right). \end{array}$$

Our survival dependent variable contains the output in the form of 0 (fatal) and 1 (alive). In NNAR modeling, the sigmoid activation function (identical to logistic regression) is used to translate a linear function that converts the probability from 0 to 1 [45]. This sigmoid activation function is of the form

(7) $$\begin{array}{c} g\left(z\right)=\frac{\text{exp}\left(z\right)}{1+\text{exp}\left(z\right)},\\ =\frac{1}{1+\text{exp}\left(-z\right)}. \end{array}$$

All modeling and forecasting were done in *R* [46].

## 3. Results and Discussion

As illustrated in Figure 2, the cumulative series of the confirmed COVID-19 cases retain a trend after detrending the data set. The new daily confirmed cases of COVID-19 series (Figure 2) can also reflect a unit root problem. In other words, the statistical properties such as mean, variance, and covariance of the original series are not constant over time. To remove this pattern from the data, we take the difference of the new daily cases. In Figure 3, the new case ACF plot illustrates a moving average (MA) pattern and the PACF plot indicates an autoregressive (AR) pattern. This, therefore, calls for the application of stationary series in further modeling and forecasting. A specific pattern in the ACF and PACF plots corresponds to a particular order of *p* and *q*. We decoupled our data set into two parts, namely, training and testing, with 90% of the data for training and 10% for testing to access the model accuracy [47].

Just as in the daily confirmed cases and cumulative confirmed cases, a similar pattern was observed in the daily confirmed deaths and cumulative confirmed deaths due to COVID-19 (Figures 4 and 5). As a result, the same modeling and forecasting procedure was applied here just as in the confirmed cases above.

The estimated ARIMA model for daily confirmed cases, possessing two autoregressive (AR) and two moving average (MA) terms as illustrated in Figure 3 and integrated of order 1, is given by

(8) $$\begin{array}{c} \hat{x}=\;-0.202x_{t-1}-0.0587x_{t-2}-0.094\;e_{t-1}-0.1014\;e_{t-2}. \end{array}$$

Moreover, the estimated ARIMA model for daily confirmed deaths, possessing two autoregressive (AR) and two moving average (MA) terms as illustrated in Figure 3 and integrated of order 1, is given by

(9) $$\begin{array}{c} \hat{x}=\;-0.869x_{t-1}-0.0919x_{t-2}-0.089\;e_{t-1}-0.579\;e_{t-2}. \end{array}$$

### 3.1. Forecast of Cumulative Confirmed Daily Cases of COVID-19 from February 19, 2022, to April 18, 2022

From Table 2, the NNAR model had RMSE and MAE values of 195.3010 and 143.5501, respectively, for the training data set. For the testing data set, the NNAR model had RMSE and MAE values of 2136.0690 and 1589.5690, respectively. The NNAR model's RSME and MAE values for both the training and testing data sets were the least among the ARIMA models and the other competing models. This shows that the NNAR model has higher forecast quality and assesses the data better than the rest of the models [48], making it the most appropriate candidate model for predicting the cumulative daily confirmed COVID-19 cases. We, therefore, used the NNAR model to predict the cumulative daily confirmed cases of COVID-19 from February 19, 2022, to April 18, 2022. The forecast value as illustrated in Figure 6 shows that the cumulative daily cases of COVID-19 in Pakistan will be 1,597,810 on April 18, 2022.

### 3.2. Forecast of Cumulative Confirmed Daily Deaths of COVID-19 from February 19, 2022, to April 18, 2022

The process for predicting cumulative deaths is identical to that for cumulative confirmed cases. From Table 3, the NNAR model had RMSE and MAE values of 10.36647 and 5.065002, respectively, for the training data set. For the testing data set, the NNAR model had RMSE and MAE values of 12.89895 and 8.009270, respectively. The NNAR model's RSME and MAE values for both the training and testing data sets were the least among the ARIMA models and the other competing models. This shows that the NNAR model has higher forecast quality and assesses the data better than the rest of the models [48], making it the most appropriate candidate model for predicting the cumulative daily deaths. We, therefore, used the NNAR model to predict the cumulative daily cases of COVID-19 from February 19, 2022, to April 18, 2022. The forecast value as illustrated in Figure 7 shows that the cumulative daily deaths of COVID-19 in Pakistan will be 32,628 on April 18, 2022.

## 4. Conclusion

The COVID-19 pandemic continues to destroy human life around the world. Almost every country throughout the globe suffered from this pandemic, forcing various governments to apply different restrictions to reduce its impact. This study used COVID-19 data in Pakistan from February 26, 2020, to February 18, 2022, as a training and testing data set to compare different time-series models. We estimated and assessed models on the training set and assessed them on the testing set. We computed the RSME and MAE for the ARIMA model, the NNAR model, and other competing models. The out-of-sample RMSE and MAE of the NNAR model were the least among all other models, indicating that the NNAR model outperforms the ARIMA model and the other competing models in terms of forecasting. That is, the NNAR model has better forecast, assessment, and quality compared to the rest of the models. Based on the NNAR forecasted values, the cumulative number of confirmed COVID-19 cases will be 1,597,810 and the cumulative deaths attributed to COVID-19 will be 32,628 on April 18, 2022. We, therefore, suggest that the NNAR model can be adopted to model and forecast COVID-19 cases and deaths as well as other time-series data just like the multigene genetic programming by Niazkar and Niazkar [49]. It is worth noting that other machine learning techniques for time-series data can be considered and used in a similar manner. As COVID-19 has prolonged for more than two years and with the prevailing virus mutation, lockdown is not a feasible solution in current circumstances. Although more than half of Pakistan's population is immunized, if the government's current immunization policy continued, the cumulative cases and cumulative deaths would decrease in the coming months. It is paramount for the Government of Pakistan to boost the immunization policy and ease restrictions to flatten the curve.

## Figures and Tables

**Figure 1:** Confirmed cumulative daily cases (a) and cumulative daily deaths (b) of COVID-19 in Pakistan from February 26, 2020 to February 18, 2022 (source: https://covid.gov.pk).

**Figure 2:** Trend of COVID-19 daily cases (a) and cumulative daily cases (b) in Pakistan from February 26, 2020, to February 18, 2022.

**Figure 3:** COVID-19 daily cases with ACF (a) and PACF (b).

**Figure 4:** Trend of COVID-19 daily deaths (a) and cumulative daily deaths (b) in Pakistan from February 26, 2020, to February 18, 2022.

**Figure 5:** COVID-19 daily deaths with ACF (a) and PACF (b).

**Figure 6:** Forecast of cumulative COVID-19 confirmed cases from February 19, 2022, to April 18, 2022.

**Figure 7:** Forecast of cumulative COVID-19 daily deaths from February 19, 2022, to April 18, 2022.

**Table 1:** Summary statistics of daily confirmed cases and deaths of COVID-19 from February 26, 2020, to February 18, 2022.

	Daily cases	Daily deaths
Minimum	0	0
Maximum	8183	313
Mean	2064	41
Median	1589	31
Lower quartile	626	10
Upper quartile	3101	62
Standard deviation	1712	37

**Table 2:** Accuracy of different time-series models for predicting COVID-19 cumulative daily cases.

Method	Source	RMSE	MAE
Mean	Training	1566.384	1309.385
	Testing	2207.310	1862.713
Drift	Training	412.2189	284.6854
	Testing	2114.5660	1713.2369
Naïve	Training	412.2303	284.5769
	Testing	2177.6843	1688.9792
Holt	Training	394.6241	277.7294
	Testing	2191.3800	1740.4823
SES	Training	394.5822	277.6888
	Testing	2180.9038	1744.2653
ARIMA order SES	Training	392.7844	275.1783
	Testing	2182.1964	1754.7370
ARIMA (2, 2, 2)	Training	392.7844	275.1783
	Testing	2182.1964	1754.7370
ARIMA auto	Training	393.0668	275.3658
	Testing	2182.9865	1760.4807
NNAR	Training	195.301	143.5501
	Testing	2136.069	1589.569

**Table 3:** Accuracy of different time-series models for predicting COVID-19 cumulative daily deaths.

Method	Source	RMSE	MAE
Mean	Training	38.17407	30.06568
	Testing	34.05141	31.50445
Drift	Training	25.76414	14.11472
	Testing	33.95330	31.50954
Naïve	Training	25.76424	14.10708
	Testing	29.07091	26.64583
Holt	Training	20.28812	11.70446
	Testing	123.38359	98.10785
SES	Training	20.27235	11.62327
	Testing	37.35009	34.89225
ARIMA order SES	Training	20.20818	11.58092
	Testing	36.33789	33.86672
ARIMA order (2, 2, 2)	Training	20.20818	11.58092
	Testing	36.33789	33.86672
ARIMA auto	Training	20.06109	11.54640
	Testing	22.33402	20.61141
NNAR	Training	10.36647	5.065002
	Testing	12.89895	8.009270

## Data Availability

The data used in this study are made up of confirmed daily cases and confirmed daily deaths of COVID-19 in Pakistan from February 26, 2020, to February 18, 2022, provided by the COVID-19 Health Platform of the Ministry of National Health Services Regulation, Government of Pakistan (https://covid.gov.pk).
